# Clinical Characteristics of Patients with Pulmonary Thromboembolism Based on Computer Statistical Analysis

**DOI:** 10.1155/2022/1112960

**Published:** 2022-02-22

**Authors:** Shaofei Wang, Ruiyi Jia, Guifen Pang

**Affiliations:** The Affiliated Hospital of Chengde Medical Collage, Chengde 067000, Hebei, China

## Abstract

In order to explore the reliable clinical characteristics of patients with pulmonary thromboembolism, this paper applies computer statistical analysis methods to the analysis of clinical characteristics of patients with pulmonary thromboembolism. Moreover, starting from the actual situation, this paper combines experiments to study the case, uses sample screening and sample processing to group samples freely, and conducts grouping reliability research through data statistics methods. After verifying the reliability of the grouping, this paper combines the samples to test the effectiveness of the computer statistical analysis method applied to the clinical characteristic analysis of patients with pulmonary thromboembolism and conducts numerical analysis in combination with the comparative analysis method. The results of the research show that the computer statistical method proposed in this paper has a good effect on the clinical characteristics of patients with pulmonary thromboembolism and meets the actual needs of clinical analysis.

## 1. Introduction

Pulmonary embolism (PE) is a general term for a group of diseases or clinical syndromes that cause various emboli to block the pulmonary artery system. It mainly includes pulmonary thromboembolism (PTE), fat embolism syndrome, amniotic fluid embolism, and air embolism. Among them, PTE is the most common type, and PE usually refers to PTE in clinical practice. PTE is a disease caused by thrombosis from the venous system or right heart that blocks the pulmonary artery or its branches. Its main clinical and pathophysiological characteristics are pulmonary circulation and respiratory dysfunction. The thrombosis of PTE mainly comes from deep vein thrombosis (DVT). DVT and PTE are essentially the same disease process in different parts and different stages. The two are collectively called venous thromboembolism (VTE). PTE is a common disease in internal medicine. Its clinical symptoms are diverse, but it lacks specificity. It can be manifested as dyspnea, chest pain, hemoptysis, syncope, cough, and irritability. However, it can also be completely asymptomatic and only discovered accidentally during the diagnosis of other diseases or autopsy. The so-called typical “triad” in clinical practice, dyspnea, chest pain, and hemoptysis, is only seen in 20% of PTE patients. The severity of different PTE patients may also be very different. Mild patients may have asymptomatic or hidden symptoms, but severe patients may experience hemodynamic instability or even sudden death.

Pulmonary thromboembolism refers to a disease caused by a thrombus from the venous system or the right heart that blocks the pulmonary artery or its branches, and its main pathophysiological and clinical features are respiratory dysfunctions and pulmonary circulatory disorders. Among them, most of the thrombosis of PTE comes from the deep veins of the lower extremities [1], and the factors that can lead to deep vein thrombosis are all predisposing factors for PTE, such as surgery, fractures, chronic heart and lung diseases, and old age. The pathophysiological characteristics of pulmonary thromboembolism depend on factors such as the size and number of thrombus, the time of successive embolization of multiple emboli, whether there are other diseases at the same time, individual response differences, and the speed of thrombolysis. The pathophysiological changes in the respiratory tract mainly include severe pulmonary ventilation/perfusion imbalance, ventilatory dysfunction, reduction of alveolar surfactant, and pulmonary infarction. The pathophysiological changes of blood circulation are mainly manifested by hemodynamic changes; that is, the increase in pulmonary circulation resistance leads to pulmonary hypertension, right heart failure, and even total heart failure. Secondly, the influence of vascular endothelial function leads to blood hypercoagulability and pulmonary vasoconstriction, and the influence of neurohumoral factors eventually leads to hypotension, shock, and sudden death [2].

The clinical symptoms of PTE can range from asymptomatic to hemoptysis and even sudden death. The main manifestation is dyspnea that is difficult to explain. Other common symptoms include cough, hemoptysis, chest pain, fever, palpitations, syncope, panic, and even a sense of dying, but most of the symptoms lack obvious specificity. The so-called “triad of pulmonary infarction,” that is, dyspnea, chest pain, and hemoptysis at the same time is only seen in less than 20.0% of PTE patients [3]. The common signs of PTE are respiratory rate, increased heart rate, decreased blood pressure, cyanosis, and wet rales or wheezing in the lungs. Moreover, most patients have no obvious specificity, and only a few cases have typical lower extremity swelling, pain, and lower extremity circumference differences. Chest X-rays and CT scans of PTE patients often manifest as pulmonary plaques and shadows, sparse surrounding lung tissue texture, pulmonary hypertension, right heart enlargement, a small amount of pleural effusion, etc., which can often be confused with other lung diseases. Typical dilation of the descending pulmonary artery (Palla sign), peripheral wedge-shaped shadow on the diaphragm (Hampton sign), and regional pulmonary blood flow reduction (Westermark sign) are only more common in pulmonary infarction. The abovementioned characteristics of PTE determine that it has more similarities with other respiratory diseases in clinical manifestations and imaging changes, especially with tuberculosis. This article attempts to describe the main clinical manifestations of patients with pulmonary thromboembolism at admission and the changes in clinical manifestations after thrombolysis or anticoagulation by observing the clinical manifestations of patients with pulmonary thromboembolism during hospitalization. Through the questionnaire survey of cured pulmonary embolism patients, the general situation of patients with pulmonary thromboembolism was understood.

Based on the above analysis, this paper analyzes the clinical characteristics of patients with pulmonary thromboembolism and starts from the actual situation to combine experiments and case studies to provide theoretical support for the subsequent diagnosis and treatment of pulmonary thromboembolism.

## 2. Related Work

Pulmonary thromboembolism (PTE) is a disease caused by thrombosis from the venous system or the right heart that blocks the pulmonary artery or its branches. Pulmonary circulation and respiratory dysfunction are its main clinical and pathophysiological characteristics [4]. Pulmonary thromboembolism is the most common type of pulmonary embolism (PE), accounting for more than 90% of all PEs, and it is usually called PE or PTE. PE has a high rate of misdiagnosis, missed diagnosis, and mortality in clinical practice. The first venous thromboembolism (VTE) in the United States every year is 100/100,000, of which about 30% develop into PE [5]. Foreign autopsy statistics have found that the missed diagnosis rate of pulmonary embolism is as high as 67%, and the misdiagnosis rate is as high as 63%. Only 1/3 of patients get a correct diagnosis during their lifetime [6]. In the United States, the number of patients who die of pulmonary embolism is as high as 50,000–200,000 each year [7].

In recent years, with the improvement of clinicians' awareness of the diagnosis of pulmonary embolism and the improvement of auxiliary examination equipment, laboratory examinations, and other technical means, the early diagnosis rate of pulmonary thromboembolism has also continued to increase, and patients have received timely treatment, which has reduced the mortality rate. As a common clinical disease, PE involves many disciplines and fields. Its clinical manifestations are complex, diverse, and atypical. It is similar to the clinical manifestations of other cardiopulmonary diseases and is easy to be misdiagnosed. In mild cases, only discomfort such as chest tightness may occur, and in severe cases, sudden death may occur. About 2.5% of PE patients have sudden death as the first symptom [8]. Dyspnea is the most common symptom of pulmonary embolism [9], and less than 30% of patients have the typical pulmonary embolism triad of “hemoptysis, chest pain, and dyspnea” [10]. There are various clinical examination methods for PE, but there is no simple, easy, specific, and accurate method to diagnose pulmonary embolism, which brings certain difficulties to the early diagnosis of pulmonary embolism. As clinicians, they should constantly strengthen their diagnosis awareness, be familiar with their risk factors, clinical manifestations, examination methods, etc., and comprehensively analyze and optimize diagnosis strategies. Only in this way can the diagnosis rate of pulmonary embolism be increased and not missed and misdiagnosed, and thus, patients can receive timely treatment, which will improve the quality of life of patients and reduce mortality.

Pulmonary embolism is the general term for a group of diseases or their clinical syndromes that cause various emboli to block the pulmonary artery and its branches, including pulmonary thromboembolism (PTE), fat embolism syndrome, amniotic fluid embolism, fat embolism, tumor embolism, and air embolism; among them, PTE is the most common type of pulmonary embolism, which refers to the clinical and pathophysiological syndrome in which thromboembolism from the venous system or the right heart blocks the pulmonary artery or its branches and causes pulmonary circulation and respiratory dysfunction [11]. Pulmonary embolism is considered to be a global medical problem because of its high morbidity and mortality. In recent years, it has attracted more and more attention from the medical community at home and abroad. Although people's awareness of pulmonary embolism continues to improve, and there have been great advances in its diagnosis and treatment, its clinical manifestations are complex and changeable and lack specificity. Because some PTE patients can present with fever, if these fever patients also have chest CT, the examination will reveal patchy shadows of the lungs, which are easily misdiagnosed as pneumonia in clinical practice, resulting in a high rate of misdiagnosis and missed diagnosis. Therefore, the differential diagnosis of PTE and pulmonary infection cannot usually be achieved through basic radiological examinations or classical laboratory examinations. In recent years, studies have found that the occurrence, development, and prognosis of PTE are closely related to changes in the body's inflammatory indicators [12]. Therefore, it is necessary to further understand the clinical characteristics of inflammatory indicators in PTE patients, improve the diagnosis awareness and differential diagnosis ability of PTE, achieve early diagnosis and treatment, and reduce the mortality of patients [13]. For more than a century, the formation of thrombosis is mainly due to the three elements of thrombosis proposed in the literature [14]: vascular endothelial cell damage, venous blood flow stasis, and blood hypercoagulability. It is still the recognized pathological basis of thrombosis. As the understanding of the common pathways and interactions between the inflammatory response and the coagulation pathway continues to deepen, more and more evidence shows that the inflammatory response of different diseases (such as venous thrombosis, septic shock, and diffuse intravascular coagulation) plays an important role in the pathogenesis of cardiovascular diseases related to thrombosis [15]. In addition, the close relationship between thrombus formation and inflammation is considered to be a pioneering extension of Virchow's triangle theory. More and more evidence shows that there are extensive and complex interactions between the inflammatory response and the coagulation system. The hypercoagulable state of the blood and the inflammatory response are mutually causal. Literature [16] found that the hypercoagulable state of the blood and the inflammatory response are mutually causal, and the inflammatory response can promote the formation of thrombus in the hypercoagulable state of the blood, and thrombosis further aggravates the inflammatory response. On the one hand, inflammation can induce the blood to become hypercoagulable; as a signal transduction molecule and an inflammatory factor, which is also an effector molecule, it not only participates in the coagulation cascade reaction, but also the adhesion molecule undergoes strict temporal expression and regulation to mediate activation. Leukocytes, platelets, and endothelial cells adhere to the process and promote the release of inflammatory mediators, attack endothelial cells, damage blood vessel walls, and initiate and promote thrombosis; on the other hand, thrombus can cause inflammatory reactions: thrombus load in the vascular cavity induces proinflammatory mediators (such as adhesion molecules and cytokines) expression and release increased, thereby further promoting local inflammation. In recent years, a large amount of literature supports this view, and the research in literature [17] supports that inflammation is involved in the formation of venous thrombosis. Literature [18] proposed that infection, especially lung infection, is considered an important predisposing factor of PTE, and the risk of PTE in patients after respiratory infection can increase by 2 to 3 times. However, in clinical practice, because some PTE patients can present with fever, if these fever patients also show patchy shadows of the lungs on the chest CT examination, they are easy to be misdiagnosed as pneumonia in the clinic. Therefore, the differential diagnosis of PTE and pulmonary infection cannot usually be achieved through basic radiological examinations or classical laboratory examinations. Therefore, finding a serological inflammatory marker that is early, highly sensitive and specific, easy to implement, and low cost to help confirm the diagnosis has become an urgent and primary problem. This article summarizes the characteristics of changes in common inflammatory indicators in patients with pulmonary embolism and methods to reduce the misdiagnosis rate and missed diagnosis rate of pulmonary embolism and improve the early recognition of pulmonary embolism patients, which will enable pulmonary embolism patients to receive a timely and correct diagnosis and treatment, which would further improve their survival rate, inflammation indicators, and pulmonary embolism.

## 3. Materials and Methods

We conducted prospective data collection on all suspected pulmonary embolism patients who met the inclusion criteria in the hospital from January 2019 to August 2021, including outpatients, emergency rooms, intensive care units, and inpatients. Moreover, we excluded cases that met the exclusion criteria, and all patients signed a written informed consent form.

### 3.1. Case Selection Criteria

1. Patients with pulmonary embolism cannot be ruled out. There are clinical symptoms such as dyspnea, chest pain, hemoptysis, and syncope.
2. The onset is within 2 months.
3. The patient is older than 18 years old.

Patients can be diagnosed if they meet any of the following 5 items: (1) CT pulmonary angiography suggests pulmonary embolism; (2) pulmonary angiography suggests pulmonary embolism; (3) pulmonary radionuclide ventilation and perfusion scans indicate that ventilation and perfusion imaging do not match and indicate pulmonary embolism, while clinical tests indicate a high probability of pulmonary embolism; (4) surgery or autopsy confirms thrombosis in the pulmonary artery; and (5) pulmonary embolism is diagnosed within three months of follow-up [19].

We use the quantitative latex agglutination method (i.e., the immunoturbidimetric method). The cutoff value refers to the diagnosis and treatment of pulmonary thromboembolism established by the Chinese Medical Association Respiratory Diseases Branch, which is 500 ng/ml, and D-dimer ≥500 ng/ml is positive.

In the dichotomy, the computer statistical analysis score <4 points is impossible and >4 points is possible. In the simple computer statistical analysis and scoring, <1 is impossible and >1 is possible. In the subjective experience score, the possibility of evaluating pulmonary embolism is 0–100%, <30% is impossible, and >30% is possible.

The patient fills in a unified form, including general conditions (gender and age), vital signs (temperature, blood pressure, heart rate, breathing, and oxygen saturation), risk factors (recent immobilization or surgery <4 weeks, previous smoking, or family history of VrE, tumor or being treated, central venous catheterization, etc.), clinical symptoms (dyspnea, chest pain, hemoptysis, syncope, lower limb pain, etc.), objective physical signs (jugular vein filling, P2 hyperactivity, dry and wet lung rales, the circumference of both lower limbs, etc.), and laboratory tests (blood routine, blood gas, D-dimer, etc.).

SPSS 15.0 software was used for statistical analysis. Common causes, symptoms, and signs are described in percentages. All data collectors have received standardized training in advance, and a doctor collects the abovementioned data. First, the patient's pulmonary embolism possibility (0.100%) is evaluated clinically based on subjective experience. Then, the computer statistical analysis scores are scored item by item, and the total score is calculated, and the patients are divided into possible groups and impossible groups. At the same time, laboratory tests such as D-dimer detection are carried out. Patients who are not able to score by computer statistical analysis and are negative for D-dimer do not need further examination and treatment and directly enter the 3-month follow-up period. For patients with possible computer statistical analysis scores or positive for D-dimer, further imaging tests are required, including pulmonary ventilation-perfusion (v/0) scan, CT pulmonary angiography (CTPA), pulmonary angiography (PAA), and lower extremity venous compression ultrasound (CUS). If the result is negative, the patient enters the 3-month follow-up period. Anticoagulant or thrombolytic therapy is given to those who are positive. Moreover, all patients who ruled out pulmonary embolism were followed up by telephone or outpatient. If the patient has any symptoms of pulmonary embolism or DVT within 3 months, the patient will be admitted to the hospital immediately for related examinations to rule out or confirm the diagnosis of pulmonary embolism. Finally, all cases are scored and grouped retrospectively using a simple computer statistical analysis score (Figure 1) [20].

## 4. Result

After excluding cases that did not meet the inclusion criteria, there was no significant difference in basic parameters between PE patients and non-PE patients. There was no significant difference between the former male and the latter male. The results are shown in Table 1. There are 8 clinical features with significant differences, namely, difficulty breathing, syncope, lower limb pain, breathing speed>20 times/min, lower limb circumference difference >l cm, near term breaking (<4 weeks), recent history of surgery (<4 weeks), and past history of VrE or family history of VrE. Compared with non-PE patients, PE patients have a higher incidence of syncope, lower limb pain, lower limb circumference difference >l cm, near term breaking (<4 weeks), recent history of surgery (<4 weeks), and previous smoking history or family history of VTE. On the contrary, non-PE patients have a higher incidence of difficulty breathing and breathing faster than 20 times/min than PE patients. The other 8 items include chest pain, hemoptysis, heart rate increase >100 beats/min, oxygen saturation <95%, jugular vein filling, P2 hypertrophy, tumors, and a history of chemotherapy and smoking. There was no significant difference between them. The results are shown in Table 2. The corresponding statistical graphs are shown in Figures 2 and 3.

We divide all patients with suspected pulmonary embolism into three groups according to their ages: <65 years old, 65–75 years old, and >75 years old, and compare the incidence of PE in each age group. The results showed that the incidence of PE is the highest in the 65- to 75-year-old group, and the incidence of PE in the <65-year-old group and the >75-year-old group was basically similar. However, no significant difference is found between the three groups. The results are shown in Table 1 and Figure 4.

AUC (area under the curve) is defined as the area enclosed by the coordinate axis under the ROC curve. Obviously, the value of this area will not be greater than 1. Since the ROC curve is generally above the line *y* = *x*, the value of AUC ranges between 0.5 and 1. The closer the AUC is to 1.0, the higher the authenticity of the detection method; when it is equal to 0.5, the authenticity is the lowest and has no application value. The receiver operating curve (ROC curve) is used to test the effectiveness of various scores in the diagnosis of pulmonary embolism, and the area under the ROC curve (AUC) is used to indicate the effectiveness. The AUC of the subjective experience score, computer statistical analysis score, and simple computer statistical analysis score are shown in Table 3 and Figures 5to 7.

This article evaluates the method proposed in this paper, that is, it evaluates the effect of the computer statistical method proposed in this paper on the clinical characteristics of patients with pulmonary thromboembolism, and the results shown in Figure 8 are obtained.

From the above research, it can be seen that the computer statistical method proposed in this paper has an effect evaluation of 94 points or more in the clinical characteristics of patients with pulmonary thromboembolism, which shows that the effect of this method is very good.

## 5. Analysis and Discussion

The clinical manifestations of PTE are complex and diverse and lack specificity. Clinically, some patients with PTE may present with nonspecific symptoms such as fever, cough, chest pain, or a small amount of pleural effusion. Therefore, because of insufficient experience or insufficient attention to PTE, clinicians often misdiagnose these patients as pulmonary infections. The results of the study showed that compared with the normal control group, the inflammation-related indicators in the blood of PTE patients increased significantly. It suggests that inflammatory reactions also exist in PTE patients, so it is often difficult to distinguish the above clinical manifestations from lung infections. Many previous studies have shown that there are many high-risk factors for the occurrence of PTE, which mainly include hereditary and acquired high risk factors. With the increasing understanding of the common pathways and interactions between inflammatory response and blood coagulation pathways, more and more evidence shows that the inflammatory response of different diseases, such as venous thrombosis, diffuse intravascular coagulation, and septic shock, plays an important role in the pathogenesis of cardiovascular diseases related to thrombosis. In the recent guidelines for the diagnosis and treatment of PTE, infection, especially lung infection, is considered to be an important predisposing factor for PTE.

In recent years, NLR, PLR, and RDW have received more and more attention as new inflammation predictors. The increase in NLR is the result of an increase in the neutrophil count and a decrease in the lymphocyte count. In recent years, it is believed that this ratio is not only a new marker for evaluating systemic inflammation, but also that the increase in the NLR ratio is closely related to the mortality of cardiovascular diseases. During the formation of PTE, severe hypoxia and acute stress caused by pulmonary artery obstruction can increase the activity of neurohormones and the adrenergic system. The thrombus load induces the release of inflammatory cytokines, prompts the rapid production of a large number of neutrophils, and accelerates the rate of lymphocyte apoptosis. At the same time, neutrophils can produce a variety of inflammatory mediators, such as oxygen free radicals, myeloperoxidase, and elastase. Moreover, a large number of inflammatory mediators can cause tissue damage to release more tissue factors, which leads to thromboembolic events and aggravates the patient's condition. Therefore, the increase in the number of neutrophils may be related to the inflammatory process leading to thrombosis.

The clinical symptoms of embolism are not specific, so the diagnosis is relatively difficult. Acute pulmonary embolism often causes chest pain and difficulty breathing. It often occurs suddenly, and it may develop gradually over several days to several weeks. Pleural pain and hemoptysis often occur in patients with pulmonary infarction, and shortness of breath and increased heart rate are also common. The signs of pulmonary hypertension include jugular venous filling, P2 hyperactivity, right ventricular galloping rhythm, and elevated right ventricular pressure. Pain and swelling of the lower limbs and increased skin temperature are often clues to the diagnosis of DVT patients. The analysis of various clinical factors showed that there were 8 significant differences in clinical features. For syncope, lower limb pain, lower limb circumference difference ≥1 cm, near term breaking (<4 weeks), recent surgical history (<4 weeks), and previous history of VrE or family history of VrE, and the incidence of pulmonary embolism is higher than that of nonpulmonary embolism patients. None of the nonpulmonary embolism patients showed syncope. The reason may be that common causes of syncope are generally related to cardiovascular and cerebrovascular diseases, which are relatively rare in respiratory patients. Therefore, patients with only syncope or concurrent cardiovascular and cerebrovascular symptoms are often not considered as pulmonary embolism first. In patients with pulmonary embolism, there is pain in the lower extremities, and the difference in the circumference of the lower extremities>1 cm accounts for about one-third.

Past history of vrE suggests that patients have predisposing factors for pulmonary embolism, and family history of vrE suggests that patients may have genetic factors for pulmonary embolism, mainly factor V mutations, protein C and protein S deficiency, and antithrombin deficiency. In this study, 3 patients with pulmonary embolism were younger than 30 years old, so there may be corresponding genetic factors. However, ordinary hospitals cannot do related examinations. If such patients have repeated emboli, lifelong anticoagulation therapy may be required for prevention. The above three items are all risk factors for pulmonary embolism, but less than half of the patients have the above manifestations. On the contrary, the incidence of dyspnea and breathing speed >20 times/min is higher in nonpulmonary embolism patients than in pulmonary embolism patients. The vast majority of nonpulmonary embolism patients have symptoms of difficulty breathing. The reason may be that screening doctors are more vigilant about respiratory symptoms and are likely to select patients with shortness of breath into the group, including those with COPD, asthma, and pneumothorax. The other 8 items include chest pain, hemoptysis, heart rate increase >100 beats/min, oxygen saturation <95%, jugular vein filling, P2 hypertrophy, tumors, chemotherapy, and smoking history, and there is no significant difference in the incidence of pulmonary embolism. The above data suggest that the clinical characteristics of pulmonary embolism are quite different, and the experience of the screening doctor also affects the judgment of pulmonary embolism. It can be seen that clinical manifestations can only indicate the possibility of pulmonary embolism, and there is insufficient evidence to diagnose or rule out pulmonary embolism by relying on certain clinical features.

## Figures and Tables

**Figure 1:** Research steps.

**Figure 2:** Epidemiological and clinical characteristics of non-PE patients.

**Figure 3:** Epidemiological and clinical characteristics of PE patients.

**Figure 4:** Histogram of PE incidence based on age difference.

**Figure 5:** Sensitivity, specificity, negative predictive value, and AUC of the subjective experience score in the diagnosis of PE.

**Figure 6:** Sensitivity, specificity, negative predictive value, and AUC of the computer statistical analysis score in the diagnosis of PE.

**Figure 7:** Sensitivity, specificity, negative predictive value, and AUC of the simple computer statistical analysis and scoring in the diagnosis of PE.

**Figure 8:** Evaluation of the effectiveness of computer statistical analysis methods.

**Table 1:** Statistics of PE incidence based on age differences.

Ages	PE incidence (%)
<65	20.70
65–75	35.10
>75	23.40
All ages	25.90

**Table 2:** Epidemiological and clinical characteristics of patients with suspected pulmonary embolism.

Parameter	Non-PE patients		PE patients		*P*
	Yes	No	Yes	No	
	65.2 ± 13.1		66.2 ± 13.5		≤005
Male	0.65	0.35	0.69	0.31	>0.05
Difficulty breathing	0.92	0.08	0.64	0.36	>0.05
Chest pain	0.34	0.66	0.47	0.53	≤005
Hemoptysis	0.21	0.79	0.25	0.75	>0.05
Syncope	0.00	1.00	0.11	0.89	>0.05
Lower limb pain	0.04	0.96	0.36	0.64	≤005
Faster breathing	0.57	0.43	3.69	-2.69	≤005
Increased heart rate	0.38	0.63	0.28	0.72	≤005
Oxygen saturation ≤95%	0.53	0.47	0.36	0.64	>0.05
The difference in circumference of lower limbs is ≥1 cm	0.07	0.93	0.28	0.72	≤005
Filling of the jugular vein	0.44	0.56	0.28	0.72	>0.05
P2 excitement	0.34	0.66	0.22	0.78	>0.05
Near term breaking (≤4 weeks)	0.17	0.83	0.44	0.56	≤005
Recent history of surgery (≤4 weeks)	0.10	0.90	0.25	0.75	≤005
Tumor or undergoing chemotherapy	0.13	0.87	0.22	0.78	>0.05
Smoking room	0.37	0.63	0.39	0.61	>0.05
Past history of VTE	0.02	0.98	0.14	0.86	≤005

**Table 3:** Sensitivity, specificity, negative predictive value, and AUC of the three scoring methods in the diagnosis of PE.

	Subjective experience score		Computer statistical analysis score		Simple computer statistical analysis and scoring	
	≤30%	>30%	≤4		≤30%	>30%
PE incidence	24.20	26.70	12.90%	PE incidence	24.20%	26.70%
Sensitivity	61.30%		72.40%		75.20%	
Specificity	42.4%		65.60%		53.90%	
Negative predictive value	76.1%		87.50%		86.60%	
AUC	0.61%		0.751		0.714	

## Data Availability

No data were used to support this study.
